# Classification and Optimization of Basketball Players' Training Effect Based on Particle Swarm Optimization

**DOI:** 10.1155/2022/2120206

**Published:** 2022-01-12

**Authors:** Quanfei Zhu

**Affiliations:** Changzhou College of Information Technology, Changzhou, Jiangsu, China

## Abstract

Since the professionalization of basketball in China, the number of teenagers participating in basketball training has gradually increased, which has promoted the improvement of basketball level in China. Teenagers ‘love' for basketball further promotes the improvement of basketball level in China. However, the reality of basketball in China still lags far behind that of developed basketball countries, in which backward training is an important aspect. This paper mainly makes a comprehensive overview of the training effect and classification of basketball players through particle swarm optimization, objectively evaluates the training effect of physical fitness, and proposes corresponding optimization measures, aiming at the scientific optimization of physical training for basketball players in China. In order to rationally arrange the training methods, control the training process, and make the training scientific, the effectiveness of the particle swarm optimization algorithm for the classification of basketball players' training effects is analyzed, and a new population-based optimization method is proposed. The experimental results verify the superiority of the particle swarm optimization algorithm. It is an inevitable choice to enhance the physical strength level of basketball reserve strength by using appropriate methods to train basketball players.

## 1. Introduction

The particle swarm optimization (PSO) algorithm is a global optimization evolutionary algorithm based on swarm intelligence [1]. The algorithm uses the speed-position search model to guide the optimization search through the group intelligence cooperation and competition between the groups, which can effectively overcome the local pole. Small problem, therefore, is a kind of promising neural network training algorithm [2]. The evolutionary algorithm has strong convergence ability, does not need to rely on the gradient information of the derivative of the problem, and uses it to train the neural network, which can improve the neural network. The generalization ability can improve the convergence speed and learning ability of the neural network [3]. Particle swarm optimization is a new evolutionary algorithm that is superior in solving multipeak problems. Particle swarm optimization (PSO) is an optimization algorithm based on swarm intelligence theory. It optimizes the search through group intelligence guided by cooperation and competition among particles in the population [4]. Compared with evolutionary algorithm, PSO has kept global search strategy based on population, but it uses speed-displacement model of simple operation, to avoid the complex genetic operation, the nonlinear function optimization, the voltage stability control, and dynamic target optimization of practical problems such as the success application [5, 6]. The speed of particle swarm optimization algorithm—displacement search model of simple operation, low calculation complexity, and global search and local search—in coordination with the inertia weight can ensure the optimal solution with the larger probability, overcome the defect of local optimal BP algorithm, and improve the convergence speed of local area, to avoid in the process of GA in local search convergence stagnation [7].

Basketball, as one of the “three big balls,” was introduced into China earlier and received a wider audience and has become one of the most popular sports [8]. Physical fitness is the most basic guarantee of basketball players' athletic ability and also the most important part of their athletic ability. Modern basketball is developing at a high speed along the direction of “high, fast, accurate, and strong.” The players are tall, but tall and not “stupid,” and the technology tends to be comprehensive [9]. In the whole match, the team emphasized attack and defense speed, rhythm, and more emphasis on the oppression of confrontation. The high-speed, strong-confrontation, and fast-paced matches made the team members' physical contact more frequent [10]. Looking at the world basketball arena, the athletes' personal physical quality is crucial. Without a good physical reserve, athletes' competitive ability is like a castle in the air and cannot be talked about [11]. The quality of basketball players' training will directly affect the future development of basketball. If we want to improve, we must pay attention to training bit by bit, laying a solid foundation for basketball players' physical fitness. Through effective physical training, we can not only grasp the sensitive period of basketball players' physical fitness, but also promote basketball players to better grasp reasonable technical movements and promote basketball players' ultimate success [12]. Scientific physical training of basketball players not only contributes to the overall development of their sports quality but also lays a foundation for improving their competitive ability. It is also a favorable guarantee for technical and tactical training and is also the direction of the development trend of modern basketball [13].

Particle swarm optimization algorithm is an evolutionary computing technology based on swarm intelligence method, introducing the concept of “group” [14]. PSO is a group-based optimization tool and an iterative optimization tool. By studying the behavior of similar biological groups, researchers find that there is a social information sharing mechanism in biological groups, which provides an advantage for the evolution of groups. PSO algorithm is inspired from the behavior characteristics of biological groups and used to solve optimization problems, which is also the basis for the formation of PSO algorithm [15]. In PSO, the potential solution of each optimization problem can be imagined as a point in the d-dimensional search space, which is called “particle.” All particles have a fitness value determined by the objective function, and the search is conducted in a population composed of such a group of random particles [16]. Each particle is based on its own flight experience and flight experience of the companions to adjust their flight. The best place each particle has experienced during the flight is the optimal solution found by the particle itself. The traditional training view is that in order to improve athletic performance, it is necessary to carry out large-volume, high-intensity training [17]. Numerous practices have proved that the improvement of the level of competition is the result of years of systematic training under the conditions of continuous training. In the training, the pursuit of large amount of exercise and high intensity will cause sports bruises, which will cause the athletes' sports potential to die prematurely. This will bring disadvantages to the improvement of the competitive level [18]. Therefore, the research on the classification and optimization of basketball players' training using particle swarm optimization algorithm is very useful for the training of basketball players. The key problems in the development of China's basketball market are the backward consciousness of market economy and the unbalanced market development, and many theoretical problems have not been completely solved. Professional basketball marketing strategy lacks foresight and long-term vision. Teenagers, the main consumer group, have not received due attention. The imperfection of the current management system and documents has affected the benign operation of China's professional basketball market.

In this paper, we propose a particle swarm optimization (PSO) algorithm, which is a new algorithm for the classification and optimization of training effect of regional basketball players.

In summary, our contributions are as follows:

1. This algorithm is an optimization algorithm based on population. Each particle in the population represents a feasible solution to the problem and has a fitness value related to the objective function.
2. This technology solves the classification and optimization of basketball players' training effects by simulating the behavior of biological groups, forms a theoretical system with swarm intelligence as the core, and makes breakthroughs in some practical application fields.
3. Fast search speed, high efficiency, and simple algorithm are provided, suitable for real value processing.

## 2. Related Work

Through observation and research on biological communities, it is found that swarm intelligence generated by complex behaviors such as cooperation and competition among individuals in biological communities can often provide efficient solutions to specific problems [19]. Kennedy and Eberhar in the United States, inspired by the foraging behavior of birds, proposed the particle swarm optimization algorithm in 1995. The original idea was to simulate simple social systems and study and explain complex social behaviors. Later, it was found that particle swarm optimization algorithm could be used to solve practical optimization problems, especially engineering optimization problems [20]. Compared with the evolutionary algorithm, PSO keeps the global search strategy based on population, but the operation of the speed-displacement model is simple and avoids the complex genetic operation. Its unique memory enables it to dynamically track the current search situation and adjust its search strategy. Compared with evolutionary algorithm, particle swarm optimization is a more efficient parallel search algorithm [21]. In 2013, some scholars proved that the larger inertia weight is advantageous to global search with particle swarm optimization, while the smaller inertia weight population is more inclined to local search through the experiment of dynamic environment multiswarm optimization based on particle swarm optimization [22].

Basketball is a big sport. Participating in basketball can enhance the physical fitness of athletes, and at the same time train their organizational ability, communication ability, and teamwork ability. In short, basketball is a very good sport. For basketball players, in order to improve their basketball skills effectively, they need to master all kinds of basketball skills. There are many methods of basketball training. In the process of training athletes, classified training methods are usually adopted [23]. In 2007, some scholars based their study on the effects of two short-term training programs on the physical and technical ability of young basketball players. Considering both innate and acquired factors, it is considered that “physical energy is the morphological structure and function obtained by the human body through congenital inheritance and acquired training, combined with the potential for regulation and its potential for material energy storage and transfer and the ability to combine with the external environment [24]. In 2010, some scholars based their research on the impact of increased load and unloaded training on the jumping ability of basketball players pointing out that the load intensity of Chinese youth men's basketball team before training is lower than the game load intensity, not because of the training time. The length and duration of intense activities are different; it is because the ratio of total time in training to the total time of training sessions is too high, and the interval time is too long after each activity [25].

## 3. Materials and Methods

Particle swarm optimization (PSO) arises from the simulation of migration and population in the process of bird foraging. Similar to genetic algorithm, PSO is also an optimization tool based on iteration. The system is initialized as a set of random solutions, and the optimal solution is searched by iteration in some way. However, PSO has no “selection,” “crossover,” and “mutation” operators of genetic algorithm, and its coding method is simpler than GA. So PSO algorithm is easy to understand and implement. It has developed rapidly in recent years and has been successfully applied in many aspects. Each particle in particle swarm optimization adjusts its flight according to its own flight experience and the flight experience of its companions. The best position each particle has experienced in the flight process is the optimal solution found by the particle itself. The best position the group has ever experienced is the best solution the group has found so far. The former is called the individual extreme value, and the latter is called the global extreme value. In practice, the fitness value determined by the optimization problem is used to evaluate the “good or bad” degree of particles. Each particle constantly updates itself through the above two extremums, thus generating a new generation of population. When solving the optimization problem of PSO, each particle remembers and follows the current optimal particle to search in the solution space. The process of each iteration is not completely random. If a better solution is found, the next solution will be found based on this. Particle swarm optimization (PSO) algorithm originated from the simulated social system, but it lacks a solid mathematical foundation.

In order to speed up the search speed in the model, a triangular distribution method is proposed. This paper analyzes the statistical law of velocity and puts forward the objective distribution probability and subjective probability. These probability distributions are reasonably simplified into easy to operate triangular distributions, and then it is analyzed that this probability method can quickly approach the target value. Through theoretical data trial calculation and comparison, its search effect is better. The particle swarm optimization algorithm uses a speed-position search model. The search for particles in the solution space based on this model is shown in Figure 1. Each particle represents a candidate solution of the solution space. The degree of the solution is determined by the fitness function. The velocity determines the displacement of the particle in the number of iterations of the search space unit. Among them, the adaptation function is defined according to the optimization goal.

Similar to chromosomes in genetic algorithm, particles in PSO are basic constituent units, representing a candidate solution of solution space. If the solution vector is set as d-dimensional variable, then when the number of algorithm iterations is *x*, the ith particle can be expressed as

(1) $$\begin{array}{c} \frac{\text{d}x_{1}^{\left(1\right)}}{\text{d}t}+ax_{1}^{\left(1\right)}=\sum_{i=1}^{N}b_{i}x_{i}^{\left(1\right)}. \end{array}$$

Particle velocity represents the change in the position of the particle in the unit iteration times, namely, the displacement of the particle in the d-dimensional space representing the solution variable, which can be expressed as

(2) $$\begin{array}{c} f\left(t\right)=\sum_{j=1}^{N}\sum_{k\in Z}d_{k}^{j}\phi_{jk}\left(t\right)+\sum_{k\in Z}c_{k}^{N}\phi_{Nk}\left(t\right). \end{array}$$

The fitness function is determined by the optimization objective, which is used to evaluate the search performance of particles and guide the search process of particle population. When the iteration stops, the optimal solution variable of the fitness function is the optimal solution of the optimal search. See Table 1 for details.

(3) $$\begin{array}{c} x_{1}^{\left(0\right)}\left(k\right)+az_{1}^{\left(1\right)}\left(k\right)=\sum_{i=2}^{N}b_{i}x_{i}^{\left(1\right)}\left(k\in K,\;K=1,2,\ldots ,n,\ldots \right). \end{array}$$

PSO is first initialized as a group of random particles (random solutions), and then the optimal solution is searched by iteration. In each iteration, the particle updates its velocity and position through individual and global extremums:

(4) $$\begin{array}{c} \hat{a}={\left(B^{T}B\right)}^{-1}B^{T}Y_{N},\\ W=\alpha \left(\beta \left(\frac{E_{i-\text{current}}^{2}}{E_{i-init}^{2}}\right)+\left(1-\beta \right)\frac{d_{i}}{d_{\text{max}}}\right), \end{array}$$

where *α* is a random number evenly distributed between (0, 1) and *ß* and *B* are learning factors.

The individual extremum is the solution with the best fitness for a single particle from the initial search to the current iteration.

(5) $$\begin{array}{c} E_{Rx}\left(l\right)=E_{Rx-elec}\left(l\right)=lE_{elec}. \end{array}$$

The global extremum is the solution with the best fitness for the entire particle population from the beginning of the search to the current iteration.

(6) $$\begin{array}{c} d_{\text{max}}=\text{max}\left\{d_{i}\right\},\\ i=1\ldots n. \end{array}$$

Particles keep tracking individual and global extremums in the solution space until they reach the required number of iterations or meet the required error criteria.

Basketball is a big sport. Learning basketball and mastering basketball skills can enhance athletes' physique. If they often participate in competitions, they can also cultivate athletes' organizational ability and communication ability and may also cultivate athletes' positive and optimistic attitude towards life. Based on the overall level, basketball is a “sunshine, can enhance physical fitness, and cultivate people's ability to cooperate” sports.

In the process of solving the practical optimization problem, the inertia weight decreases linearly with the number of iterations. In the initial stage of the search, particle swarm can search the whole solution space with a large probability and can quickly converge to the local region where the optimal solution is. Then, with the decrease of inertia weight, the particle population can achieve local fine-tuning in this region. In the process of convergence, the number of particles is gradually reduced to improve the particle efficiency. The increasing phase in the periodic oscillation term represents the random emergence of new particles to increase the diversity of particle swarm. The particle swarm optimization algorithm with a large inertia weight has a strong global search ability, while the algorithm tends to local search if the inertia weight is small. The formula is shown in (7) and (8), and the graph is shown in Figure 2.

(7) $$\begin{array}{c} E\left[d_{to\text{ CH}}^{2}\right]=\iint {\left(x^{2}+y\right)}^{2}\rho \left(x,y\right)\text{d}x\text{d}y \end{array}$$

(8) $$\begin{array}{c} E\left[d_{to\text{ CH}}^{2}\right]=\frac{1}{2\pi }\frac{M_{1}*M_{2}}{k}. \end{array}$$

The convergence factor may be used to ensure convergence of the particle swarm optimization algorithm. The convergence factor model is as follows:

(9) $$\begin{array}{c} k=\sqrt{\frac{\xi_{fs}}{\xi_{\text{amp}}}}\sqrt{\frac{M_{1}M_{2}N}{2\pi }}\frac{1}{d_{to\;BS}^{2}}. \end{array}$$

The particles to be crossed are finally selected from all the examples with a certain crossover probability and then randomly combined to perform the cross operation to produce the descendant particles. The position and velocity vectors of the descendant particles are as follows:

(10) $$\begin{array}{c} E_{\text{non}-\text{CH}}=lE_{elec}+l\xi_{fs}\frac{1}{2\pi }\frac{M_{1}M_{2}}{k},\\ E_{\text{cluster}}=E_{\text{CH}}+\left(\frac{N}{k}-1\right)E_{\text{non}-\text{CH}}\approx E_{\text{CH}}+\frac{N}{k}E_{\text{non}-\text{CH}}. \end{array}$$

Sports quality includes strength, speed, endurance, agility, and flexibility. It is not only the functional ability of human body in the process of completing the movement, but also the basis of mastering other competitive abilities. It is of great significance to the selection and training of basketball players. Basketball is a comprehensive and competitive sport. Any sport quality should not be neglected. Especially the upper limb strength and speed endurance which are easy to show are particularly important. The key to improving athletes' physical fitness lies in the harmonious and unified level of load stimulation and functional adaptation. Therefore, physical training can effectively improve the shape and function of human body according to the type of load stimulation applied. This load stimulation is what sports need. The effect of athletes' training is to make their body adapt to the external environment constantly, break the original biological adaptation and balance of the body, and achieve a new stable state after a period of adaptation under the condition of meeting the physical ability required by the fierce competition. The particle swarm optimization algorithm is an optimization algorithm based on swarm intelligence theory, which guides the optimization search through the group intelligence generated by the cooperation and competition among the particles in the group. Compared with evolutionary algorithms, PSO retains a population-based global search strategy, but its speed-displacement model is simple to operate and avoids complex genetic operations. The velocity-displacement search model of particle swarm optimization algorithm is simple in operation and low in computational complexity and coordinates global search and local search through inertia weight. Inertia weight is an important parameter to balance the ability of global search and local search in particle swarm optimization algorithm. It is necessary to adopt dynamic adaptive inertia weight strategy based on different dimensions of different particles in the early stage of evolution to speed up the convergence speed. In the later stage of evolution, the linear decreasing weight strategy is adopted. At the same time, in order to prevent falling into local optimization, chaotic variation is introduced in time to increase population diversity. It can guarantee the optimal solution with a large probability and overcome the local optimal defect of BP algorithm. It can also improve the convergence speed of local regions and avoid the convergence and stagnation of GA in the local region search process.

## 4. Results

Particle swarm optimization (PSO) is a problem in which individuals search for the optimal solution through cooperation and competition. Movement speed refers to the body's ability to move quickly over a certain distance. The distance a player moves quickly on a basketball court is usually less than 30 meters. Response speed refers to the human body's ability to respond quickly to various signal stimuli. Reaction speed is the premise for athletes to make all kinds of actions. The training can adopt the methods of using signals and moving targets, such as shadow training, three people passing two balls, the coach sending signals, and the athletes responding to the requirements. Flexibility refers to the range of motion of the joints and the elasticity and extension of the ligaments, tendons, muscles, skin, and other tissues across the joints. Flexibility plays an obvious role in promoting the overall development of physical fitness. We should make full use of the development of flexibility in childhood to achieve twice the result with half the effort. The main training methods are active exercises, such as using the arch and step pressure of ribs, positive pressure, back pressure, swing legs, shoulder pressure, body lateral extension, in situ flexion of fingers, wrists, body forward bending, and supine leg raising. Attention should be paid to the alternation of flexibility exercises in different parts. Sensitivity refers to the ability of the human body to complete movements quickly, coordinately, agilely, and accurately under various changing conditions. Sensitivity quality is determined by the flexibility of cerebral cortex nerve process. High flexibility of athletes' cerebral cortex nerve can make muscles contract quickly and relax in time. The action rhythm is fast and coordinated. The degree of flexibility training of cerebral cortex nerve process will determine the level of sensitivity quality.

Many practical engineering problems are essentially function optimization problems or can be transformed into function optimization problems. For function optimization, there are some mature solutions such as genetic algorithms. However, for complex functions with ultra-high dimensional and multilocal extremum, genetic algorithms tend to achieve the desired requirements in terms of optimization convergence speed and accuracy. The particle swarm optimization algorithm can achieve better optimization results than the genetic algorithm when solving some typical function optimization problems. This shows that the particle swarm optimization algorithm also has a good application prospect in solving practical problems. PSO is a potential neural network training algorithm. PSO search speed is faster and can get better optimization results, which overcomes the shortcomings of the above two algorithms. In practical application problems, such as using PSO algorithm to train neural network for medical diagnosis, a high success rate has been achieved. It is now being extended to more applications. Therefore, particle swarm optimization (PSO) is used to study the classification and optimization of basketball players' training. Basketball is an antagonistic sport. Due to the restriction of opponents, it is necessary to flexibly change the direction, speed, and body posture according to the complex situation of the game at all times, which puts forward a high demand for sensitive quality.

Particle swarm optimization (PSO) algorithm has relatively good performance in training classification and optimization of basketball players and has good convergence. See Table 2 and Figures 3 and 4 for details.

PSO also verifies the redundant connection effect, the performance of the neural network, and information processing capacity surplus leading to overtraining problem. Through the result the experiment can launch, particle swarm optimization algorithm is compared with genetic algorithm and the training time approaches, and classification performance has improved significantly. If we have the same error goal, using particle swarm optimization algorithm convergence training required for the number of iterations is decreased obviously. It can be seen that the particle swarm optimization algorithm not only greatly improves the convergence speed of training, but also significantly enhances the performance of the trained neural network. The range of heart rate changes in the regular training class is large, showing the high and low staggered phenomenon; the training course reaches the highest peak. It takes a long time, the speed and slope of the heart rate curve are relatively insignificant, and the heart rate game is just the opposite, as shown in Figure 5 and Table 3.

There was no significant difference in recovery between the end of the three minutes, although there was a significant difference in heart rate before the end of the training (see Table 4). The problem of classification and optimization of basketball players' training can better reflect the contents of this paper (see Table 5).

Training is a systematic and comprehensive work, which contains a wide range of content. In order to achieve the ideal competitive ability, only the implementation of systematic principles can help, starting from weak links, from the content of training arrangements and action specifications. The training classification of basketball players using PSO is compared with that before and after optimization as shown in Figure 6. The convergence curve of PSO under different training loads is shown in Figure 7.

Testing can help athletes and coaches diagnose physical fitness, find weak links, achieve training goals, or tap potential. This is in order to change the declining trend of China's professional basketball training quality year by year as soon as possible, reverse the phenomenon of “three deficiencies” (training, management, and culture), improve the competitive ability level of professional teams and their reserve talents, shorten the gap with international strong teams, and make basketball programs contribute to the realization of a strong sports country at an early date. In basketball training, the effect will be affected in the training process, and some athletes may appear more in the subjective training content. Especially in the content of endurance training, training often leaves space for yourself. This situation has formed a certain degree of misleading after coach training and also led to the unsatisfactory effect of basketball training.

## 5. Conclusions

Due to the constraints of the system and other factors, the training period is short, the regular physical training begins relatively late, the training time is tight, the physical training is not comprehensive enough, and there is a lack of systematic training control and scientific training load, resulting in lowering the physical development level of basketball players. With a certain lag, the training effect is not obvious. For male basketball players who have not systematically practiced core strength and physical stability, short-term concentrated training can effectively improve related ability, factors that restrict the development of basketball players' physical fitness, except for the interference of factors such as the arrangement of training means. The psychological factors of the athletes in the training implementation phase are also crucial. In the formulation of physical fitness training programs for young athletes, the level and characteristics of athletes are fully considered. Particle swarm optimization algorithm is used to create an environment suitable for the development of athletes, highlight personalized training prescriptions, and effectively enhance competitive ability. While classifying and optimizing basketball players scientifically and systematically, we should lay particular emphasis on giving priority to development and combining comprehensiveness with priority to development.

## Figures and Tables

**Figure 1:** Particle swarm optimization algorithm flow.

**Figure 2:** Comparison of particle swarm optimization algorithm and time prediction.

**Figure 3:** Error evolution curve of particle swarm optimization algorithm.

**Figure 4:** Training error curve with iteration times.

**Figure 5:** Diagram of changes in heart rate of training sessions and competitions.

**Figure 6:** Comparison of basketball players' training classification and optimization before and after training.

**Figure 7:** Convergence curve of particle swarm optimization under different training loads.

**Table 1:** Performance comparison of particle swarm optimization algorithm.

	PSO
Accuracy of training samples	83.8%
Training sample error	6.76
Test sample correctness rate	81.34%
Test sample error	5.49

**Table 2:** Performance of particle swarm optimization.

Performance index	Iris	Ionosphere	Breast cancer
Error index	1.58	2.37	0.49
Classification accuracy	93.39%	94.76%	99.5
Connection number	52	513	119

**Table 3:** Basketball players' competition activities.

	Average heart rate (times/10 seconds)	Sports density (%)
*T*	4.55	2.47
*P*	<0.05	<0.08

**Table 4:** Comparison of heart rate recovery after different intensity training.

	People	Before training	End of training	Difference
Upper middle strength	43	11.49	8.54	2.95
Mid-low strength	37	5.27	3.61	1.66

**Table 5:** Statistical evaluation results.

Validity	Effective	More effective	Invalid
Frequency	7	3	1
Percentage	35	15	5

## Data Availability

The data used to support the findings of this study are included within the article.

## References

[1] Xiaoyan S., Huaixia L., Shuijuan Y. U. (2013). Short-time load prediction based on support vector machine optimized by catfish particle swarm optimization algorithm. *Computer Engineering & Applications*.

[2] Oguzhan Y (2016). Hematologic effects of enzyme Q10 supplements on basketball players applying combined training program. *The Anthropologist*.

[3] Hung J.-C. (2015). Robust Kalman filter based on a fuzzy GARCH model to forecast volatility using particle swarm optimization. *Soft Computing*.

[4] Yilmaz G. (2014). The effects of power, speed, skill and anaerobic capacity of different training models in young male basketball players. *The Anthropologist*.

[5] Jiangfu L., Lina T., Cuiping W., Tong X (2014). Measuring and calibrating extended neighborhood effect of urban cellular automata model based on particle swarm optimization. *Progress in Geography*.

[6] Kundu S., Jha A., Chattopadhyay S., Sengupta I., Kapur R. (2014). Framework for multiple-fault diagnosis based on multiple fault simulation using particle swarm optimization. *IEEE Transactions on Very Large Scale Integration Systems*.

[7] Assarzadeh Z., Naghsh-Nilchi A. (2015). Chaotic particle swarm optimization with mutation for classification. *Journal of Medical Signals & Sensors*.

[8] Zhang Y., Gong D., Hu Y., Zhang W., KIM S (2015). Feature selection algorithm based on bare bones particle swarm optimization. *Neurocomputing*.

[9] An L. B., Seok K. B., Seok K. M., YOUN K. K (2014). Electrical resistance imaging of two-phase flow with a mesh grouping technique based on particle swarm optimization. *Nuclear Engineering and Technology*.

[10] Zhang H., Jin Y. (2017). Particle swarm cooperative optimization algorithm based on geometric algebra. *Journal of Discrete Mathematical Sciences and Cryptography*.

[11] González-Bono E., Salvador A., Serrano M. A., Moya-Albiol L. (2002). Effects of Training Volume on Hormones and Mood in Basketball Players. *International Journal of Stress Management*.

[12] Shijie Y., Dan L., Qingbiao Z. (2013). Coal consumption prediction based on LSSVM optimized by Catfish Particle Swarm Optimization algorithm. *Computer Engineering & Applications*.

[13] Liu Y., Zheng X., Wang B., Zhou S., Zhou C. (2016). The optimization of DNA encoding based on chaotic optimization particle swarm algorithm. *Journal of Computational and Theoretical Nanoscience*.

[14] Asadi A. (2013). Effects of in-season short-term plyometric training on jumping and agility performance of basketball players. *Sport Sciences for Health*.

[15] Xuezhong Q., Jing L. I., Wei S. (2013). Improved fuzzy clustering algorithm based on particle swarm optimization. *Computer Engineering & Applications*.

[16] Aoki M. S., Ronda L. T., Marcelino P. R. (2017). Monitoring training loads in professional basketball players engaged in a periodized training program. *The Journal of Strength & Conditioning Research*.

[17] Notarnicola A., Maccagnano G., Tafuri S., Pesce V, Digiglio D, Moretti B (2014). Effects of training on postural stability in young basketball players. *Muscles Ligaments Tendons J*.

[18] Santos E. J., Janeira M. A. (2009). Effects of reduced training and detraining on upper and lower body explosive strength in adolescent male basketball players. *The Journal of Strength & Conditioning Research*.

[19] Czuba M., Zając A., Maszczyk A. (2013). The effects of high intensity interval training in normobaric hypoxia on aerobic capacity in basketball players. *Journal of Human Kinetics*.

[20] Ahmed T. (2013). The effect of upper extremity fatigue on grip strength and passing accuracy in junior basketball players. *Journal of Human Kinetics*.

[21] Adorable L. V., Caparino C. A. D., Abbu C. C. (2013). The effect of plyometric training on the vertical leap of university varsity basketball players. *PM&R*.

[22] Yazdani D., Nasiri B., Sepas-Moghaddam A., Meybodi M. R. (2013). A novel multi-swarm algorithm for optimization in dynamic environments based on particle swarm optimization. *Applied Soft Computing*.

[23] Tsimachidis C., Patikas D., Galazoulas C., Bassa E., Kotzamanidis C. (2013). The post-activation potentiation effect on sprint performance after combined resistance/sprint training in junior basketball players. *Journal of Sports Sciences*.

[24] Bogdanis G. C., Ziagos V., Anastasiadis M., Maridaki M. (2007). Effects of two different short-term training programs on the physical and technical abilities of adolescent basketball players. *Journal of Science and Medicine in Sport*.

[25] Khlifa R., Aouadi R., Hermassi S. (2010). Effects of a plyometric training program with and without added load on jumping ability in basketball players. *The Journal of Strength & Conditioning Research*.

